The article "SC-Dynamic R-CNN: A Self-Calibrated Dynamic R-CNN Model for Lung Cancer Lesion Detection" was published in 2022. Journal: Comput Math Methods Med.

# SC-Dynamic R-CNN: A Self-Calibrated Dynamic R-CNN Model for Lung Cancer Lesion Detection

**DOI:** 10.1155/2022/9452157

**Published:** 2022-03-28

**Authors:** Xun Wang, Lisheng Wang, Pan Zheng

**Affiliations:** ^1^China University of Petroleum, China; ^2^University of Canterbury, New Zealand

## Abstract

Lung cancer has complex biological characteristics and a high degree of malignancy. It has always been the number one “killer” in cancer, threatening human life and health. The diagnosis and early treatment of lung cancer still require improvement and further development. With high morbidity and mortality, there is an urgent need for an accurate diagnosis method. However, the existing computer-aided detection system has a complicated process and low detection accuracy. To solve this problem, this paper proposed a two-stage detection method based on the dynamic region-based convolutional neural network (Dynamic R-CNN). We divide lung cancer into squamous cell carcinoma, adenocarcinoma, and small cell carcinoma. By adding the self-calibrated convolution module into the feature network, we extracted more abundant lung cancer features and proposed a new regression loss function to further improve the detection performance of lung cancer. After experimental verification, the mAP (mean average precision) of the model can reach 88.1% on the lung cancer dataset and it performed particularly well with a high IoU (intersection over union) threshold. This method has a good performance in the detection of lung cancer and can improve the efficiency of doctors' diagnoses. It can avoid false detection and miss detection to a certain extent.

## 1. Introduction

Cancer is the second leading cause of human death in the world, and its mortality and morbidity are increasing year by year. According to the data of the World Health Organization (WHO), cancer has led to 9.6 million deaths in 2018 and lung cancer ranks first, with 1.76 million deaths [1]. Compared with other cancers, the biological characteristics of lung cancer are very complex and it has a short onset time and high malignancy, which makes lung cancer still the number one “killer” of cancer [2, 3]. The main reason for the high morbidity and mortality is that the diagnosis and treatment methods of lung cancer are still at an early stage, so it is urgent to refine and improve the diagnosis methods of lung cancer.

At present, histopathological examination is the standard for pathological diagnosis of tumors, which can only be performed on tissue specimens such as surgical resection or needle biopsy. However, the tissue specimens obtained are invasive and susceptible to specimen sampling. To assist diagnostic doctors in their work and improve the efficiency of cancer diagnosis, the computed tomography (CT) [4] has been widely used in the intelligent diagnosis of medical images, becoming a powerful tool to comprehensively capture the characteristics of cancer. Computer-aided detection systems are mostly machine learning algorithms such as support vector machines, which are usually used to detect and classify tumors [5, 6]. However, they are usually limited by the assumptions made during the definition of elements and still have drawbacks such as a complex process, parameter setting based on experience, and strong dependence. For example, lung cancer detection results depend on the quality of segmentation results and the effectiveness of extracted features.

The article "SC-Dynamic R-CNN: A Self-Calibrated Dynamic R-CNN Model for Lung Cancer Lesion Detection" was published in 2022. Journal: Comput Math Methods Med.

In recent years, artificial neural networks, especially deep neural networks, have made remarkable achievements in many fields of intelligent medicine [7–9]. This learning algorithm is driven by big data, excavates rules from a large amount of data, and then classifies and judges unknown phenomena [10–16]. The continuous accumulation of medical data provides powerful materials and tools for intelligent screening and diagnosis of cancer. Zhang et al. [17] used a convolutional neural network to extract deep features and combine them with shallow features to achieve the classification of ovarian cancer. In addition, Wu et al. [18] used the deep convolutional neural network based on AlexNet to realize the classification of ovarian cancer pathological images and the accuracy rate of the model achieved 78.2%. Tajbakhsh and Suzuki [19] used an artificial neural network and convolutional neural network to test the benign and malignant classification of pulmonary nodules in CT images, and the experiment found that the performance of the convolutional neural network was better than the other types of artificial neural network in the lung lesion and tumor classification task.

With the development of the field of intelligent medical treatment, the types of diseases are increasing and the complexity of the pathological relationship between diseases is also increasing, so the requirements of a deep neural network are more and more strict. At present, mainstream object detection algorithms in deep learning are mainly based on two types: the first is a one-stage detection algorithm, which includes Yolo [20] and RetinaNet [21]; the performances of those methods are fast yet not accurate. As a representative of the one-stage algorithm, the Yolo series runs fast. It divides an image into multiple cells of the same size, predicts the category of each cell, and gives the category confidence of the bounding box. The other is a two-stage object detection algorithm, such as Fast R-CNN [22], Faster R-CNN [23], and Mask R-CNN [24]. The first stage of this algorithm takes the CT image as the input and generates the region of interest through the algorithm. The second stage is to use the output of the first stage to further classify and regress the bounding box. Although the detection accuracy of the two-stage object detection algorithm is better than the one-stage object detection algorithm, high-quality samples contribute significantly less to the network during the training process. Zhao et al. [25, 26] proposed a Cascade R-CNN network based on Faster R-CNN to solve the problem that high-quality samples contribute less to training in object detection. Through the Cascaded R-CNN network, each R-CNN network is set with different IoU thresholds. In this way, the accuracy of each network output has been improved to a certain extent and the output of the previous R-CNN network can be used as the input of the next high-precision network. Finally, the accuracy of the network will gradually improve. In addition, in order to solve the imbalance of object detection in the training process, Pang et al. [27] proposed a Libra R-CNN network, which paid attention to the problems of the sample layer, feature layer, and target layer, and balanced the imbalance through the overall balanced design. Zhang et al. [28] drew lessons from the idea of Cascade R-CNN and proposed Dynamic R-CNN, which further solved the problem of inconsistencies between training processes.

The article "SC-Dynamic R-CNN: A Self-Calibrated Dynamic R-CNN Model for Lung Cancer Lesion Detection" was published in 2022. Journal: Comput Math Methods Med.

In addition to the network's architecture, the quality of feature map extraction also greatly affects the accuracy of object detection. In most computer vision tasks, it is helpful to establish a long-distance dependency mechanism for feature map extraction. One way to model remote dependencies is to use a spatial pool or convolution operator with a large kernel window. Some typical examples, such as PSPNet [29], employ multiple spatial pool operators of different sizes to capture multiscale contexts. There is a lot of work [30–32] using a large convolution kernel or extended convolution for long-term context aggregation. By introducing an adaptive response calibration operation, SCNet [33] constructs multiscale feature representation in the building block and greatly improves the prediction accuracy.

In this study, the histologic types of lung cancers that we are looking at are adenocarcinoma, squamous cell carcinoma, and small cell carcinoma. The first two types are the major types of lung cancer of non-small cell lung cancer (NSCLC) which takes 85% to 90% of all lung cancer cases. Small cell carcinoma constitutes 10% to 15% of lung cancers [34]. The percentage of different lung cancer types objectively causes the imbalance of the image data collected. Some data preprocessing procedure is conducted to resolve its impact on our SC-Dynamic R-CNN development. The types of lung cancers studied in this research bear high-level significance and real-life value in medical practices.

The article "SC-Dynamic R-CNN: A Self-Calibrated Dynamic R-CNN Model for Lung Cancer Lesion Detection" was published in 2022. Journal: Comput Math Methods Med.

To improve the detection accuracy of lung cancer, a new lung cancer detection algorithm based on Dynamic R-CNN [28] is proposed in this paper. We divide the collected datasets into three categories: adenocarcinoma, squamous cell carcinoma, and small cell carcinoma, and amplified the data of squamous cell carcinoma and small cell carcinoma by an oversampling method. Next, we implement the SCNet [33] module into the Dynamic R-CNN network, which can fully extract lesion features. In addition, we propose a new loss function, DBS L1 loss, which further improves the contribution of high-quality samples to training. After experimental verification, we found that our algorithm has a great improvement in the detection of lung cancer compared with other advanced algorithms.

## 2. Materials and Methods

### 2.1. Materials

This paper's dataset was taken from the Shandong Provincial Hospital and Shandong Provincial Third Hospital in Shandong, China. The datasets include 34056 pathological images on 261 patients, and the lesion location was marked by professional radiologists. According to the radiologist's annotation, we selected 3442 images of lung cancer with lesions.

The data selected are firstly divided into three categories, namely, adenocarcinoma, squamous cell carcinoma, and small cell carcinoma. In this paper, we use “Adenocarcinoma,” “Squamous carcinoma,” and “small cell carcinoma” to represent these three categories. Among the pathological types of lung cancer, adenocarcinoma is the most common and there is little data on other types of cancer, which leads to the imbalance towards the number of samples of different types of lung cancer. The dataset of lung cancer is distributed as follows:

Figure 1 shows that there are 2273 samples of adenocarcinoma, 845 samples of squamous carcinoma, and 324 samples of small cell carcinoma. To more objectively train the method, we would like to have the datasets of different cancer types in a similar size; hence, for the small size of cancer-type datasets, we expanded the size of the dataset by oversampling methods. It is noticeable that the number of adenocarcinoma data samples is about three times of squamous carcinoma and eight times of small cell carcinoma, and therefore, the latter two minority class datasets were oversampled 3 times and 8 times of their original size to match the majority class, i.e., adenocarcinoma.

The article "SC-Dynamic R-CNN: A Self-Calibrated Dynamic R-CNN Model for Lung Cancer Lesion Detection" was published in 2022. Journal: Comput Math Methods Med.

Different from conventional oversampling approaches, e.g., random oversampling and synthetic minority oversampling technique (SMOT), for image data, we can synthesize samples using image processing techniques, e.g., spatial transformation including flipping, shearing, and rotating [35], gamma transformation, histogram equalization, and other methods to enhance the dataset [36]. An example of an image enhancement result is shown in Figure 2.

### 2.2. Methods

We present the next new method for robust lung cancer lesion detection in CT studies that uses Dynamic R-CNN trained on our dataset. To achieve accurate detection of lung cancer lesions, we use Dynamic R-CNN as the baseline network and use the self-calibrated convolutions to replace the traditional convolution. Besides that, we proposed a new regression loss function which is better than the loss function in Dynamic R-CNN.

We first present an overview of the method and then describe in detail its components. To make the paper self-contained, we describe all steps of the extended method.

#### 2.2.1. Model

Figure 3 shows the flow diagram of our method. The structure of the SC-Dynamic R-CNN network is similar to Faster R-CNN [23]. It is composed of two modules. The first module is a deep fully convolutional network that proposes regions, which is called the region proposal network (RPN) module. The RPN module is aimed at detecting multiple objects in a single image. The second module is the detector that uses the proposed regions, namely, Box_Head. After the Box_Head, there are two loss functions: classification loss function and regression loss function. But unlike Faster R-CNN [23], SC-Dynamic R-CNN can adjust the label assignment criteria and the shape of regression loss function automatically during training that makes better use of the training samples. In order to enhance the ability of feature representation of lung cancer, SC-Dynamic R-CNN adds SCNet [33] to the RPN module. Except that, the loss function of Dynamic R-CNN has been optimized for getting a better detection result of lung cancer.

As shown in Figure 3, initially, the lung cancer images are resized to 512 × 512 pixels for the training phase. The resize images are subsequently fed to the region proposal network (RPN) to get the proposed region. Next, the proposed regions are classified and regressed by the Box_Head module. Eventually, the classification and regression results are fed into the corresponding loss function and as the parameter update of the network. We use softmax loss as the classification loss, and regression loss uses our newly proposed loss function, the details of which will be described in the next section.

The article "SC-Dynamic R-CNN: A Self-Calibrated Dynamic R-CNN Model for Lung Cancer Lesion Detection" was published in 2022. Journal: Comput Math Methods Med.

To better exploit the dynamic property in the training stage, SC-Dynamic R-CNN uses a lower IoU threshold to better accommodate these imperfect proposals in the second-stage training (Figure 3(a)). As the training goes, the quality of proposals is continuously improved. Therefore, we can increase the threshold to better use them to train a high-quality detector, so the network can be more discriminative at higher IoU. Dynamic label assignment can be formulated as follows:

(1) $$\begin{array}{c} \text{Label}=\left\{\begin{array}{cc} 1, & \text{if }\max\text{ IoU}\left(b,G\right)\geq T_{\text{now}},\\ 0, & \text{if }\max\text{ IoU}\left(b,G\right)<T_{\text{now}}, \end{array}\right. \end{array}$$

where *T*_now_ stands for the current IoU threshold. In order to realize the dynamic property that the distribution of proposals changes over time during the training process, the dynamic label assignment will automatically update based on the proposal's statistics. Specifically, SC-Dynamic R-CNN first calculates the IoUs *I* between the proposals and its target ground truth and then selects the maximum value of *K*_*I*_ from *I* as the threshold *T*_now_. As the training goes, the IoUs *I* between the proposal and its target ground truths will increase gradually and so does the updated threshold *T*_now_.

In addition, according to the conclusion of Dynamic R-CNN [28], with the improvement of IoU threshold, the quality of positive samples will be further improved. As a result, the contribution of high-quality samples will be further decreased, which will greatly limit the overall performance. Based on the method of Dynamic R-CNN, we have improved its regression loss function and obtained more accurate results which are described in the next section.

#### 2.2.2. DBS L1 Loss

According to the conclusion of Dynamic R-CNN [28], with the improvement of the sample quality, its contribution will gradually decrease. As a result, Dynamic R-CNN adds a factor *α* based on the Smooth L1 loss function. The network adjusts the loss function by adjusting the value of the factor *α*. With the increase of factor *α*, the gradient of high-quality sample training will increase gradually, so the contribution to the network will be increased. The regression loss function of Dynamic R-CNN is shown as follows:

(2) $$\begin{array}{c} \text{DSL}\left(x,\alpha_{\text{now}}\right)=\left\{\begin{array}{cc} \frac{0.5{\left|x\right|}^{2}}{\alpha_{\text{now}}}, & \text{if}\left|x\right|<\alpha_{\text{now},}\\ \left|x\right|-0.5\alpha_{\text{now}}, & \text{otherwise}, \end{array}\right. \end{array}$$

where the *α*_now_ will decrease with the training, as shown in Figure 2.

The article "SC-Dynamic R-CNN: A Self-Calibrated Dynamic R-CNN Model for Lung Cancer Lesion Detection" was published in 2022. Journal: Comput Math Methods Med.

But the loss function can be further improved. Taking Libra R-CNN [27] as a reference, we improve the Dynamic R-CNN loss function and further improve the contribution of high-quality samples to training. The improved DBS L1 loss can be formulated as follows:

(3) $$\begin{array}{c} \text{DBSL}\left(x,\alpha_{\text{now}}\right)=\left\{\begin{array}{cc} \frac{\alpha_{\text{now}}}{b}\left(b\left|x\right|+1\right)\ln\left(b\left|x\right|+1\right)-\alpha_{\text{now}}\left|x\right|, & \text{if }\left|x\right|<\alpha_{\text{now}},\\ \left|x\right|+C, & \text{otherwise}. \end{array}\right. \end{array}$$

where *b* and *C* are constants and their values are constrained by the factor *α*.

Similar to the dynamic label assignment process in Dynamic R-CNN [28], DBS L1 loss first obtains the regression label *E* between proposals and their target ground truths. Then, we select the *K*_*α*_ minimum value from *E* to update the factor *α* in the equation.

As shown in Figure 4, with the continuous reduction of factors in DBS L1 loss, the contribution of high-quality samples to training increases gradually. Clearly, the DBS L1 loss is superior to DS L1 loss, which greatly improves the recognition accuracy of lung cancer lesions.

#### 2.2.3. Self-Calibration

Conventional 2D convolution is still used to calculate the convolution in Dynamic R-CNN [28]. But in conventional 2D convolution, each output feature map is generated by the same formula, which results in the convolutional filters learning similar patterns. In addition, the fields of view for each spatial location in the convolution feature transformation can only be controlled by the size of the predefined convolution kernel. As a result, the discrimination of the lung cancer feature map will be decreased. In order to enhance the ability of feature representation of lung cancer lesions and identify lung cancer lesions more accurately, SCNet [33] is used in SC-Dynamic R-CNN instead of traditional 2D convolution.

As shown in Figure 5, the shape of the given group of the filter is (*C*, *C*, *k*_*h*_, *k*_*w*_), where *C* is the number of channels and *k*_*h*_ and *k*_*h*_ are the spatial height and width, respectively. SCNet first separates it into four portions, each of which is responsible for different functionality. The separated filter is expressed by {*K*_*i*_}_*i*=1_^4^, and the size of each filter is (*C*/2, *C*/2, *k*_*h*_, *k*_*w*_). The input *X* will be divided into two parts before entering the self-calibrated convolutional network, which represents by *X*_1_ and *X*_2_, where *X*_1_ will conduct self-calibration through {*K*_2_, *K*_3_, *K*_4_} to produce *Y*_1_. At the same time, *X*_2_ will be manipulated by *K*_1_ and produce *Y*_2_. Finally, *Y*_2_ will be connected to *Y*_1_ to generate the final output *Y*.

The article "SC-Dynamic R-CNN: A Self-Calibrated Dynamic R-CNN Model for Lung Cancer Lesion Detection" was published in 2022. Journal: Comput Math Methods Med.

In order to collect the context information of each spatial location effectively, SCNet conducts convolution feature transformation in two different scale spaces. Firstly, input *X*_1_ will be performed with average pooling operation:

(4) $$\begin{array}{c} T_{1}=\text{AvgPool}\left(X_{1}\right). \end{array}$$

Then, the obtained *T*_1_ maps the intermediate references from the small-scale space to the original feature space by a bilinear interpolation operator. The specific formula is as follows:

(5) $$\begin{array}{c} X_{1}^{\prime }=\text{Up}\left(F_{2}\left(T_{1}\right)\right)=\text{Up}\left(T_{1}*K_{2}\right), \end{array}$$

where “∗” denotes convolution and Up (·) is a bilinear interpolation operator. The calibration operation can be formulated as follows:

(6) $$\begin{array}{c} Y_{1}^{\prime }=F_{3}\left(X_{1}\right)\cdot \sigma \left(X_{1}+X_{1}^{\prime }\right), \end{array}$$

where *F*_3_(*X*_1_) = *X*_1_∗*K*_3_, “·” denotes element-wise multiplication, and *σ* is the sigmoid function. After the calibration operation, *Y*′_1_ needs to be operated by the following formula to get the final output:

(7) $$\begin{array}{c} Y_{1}=F_{4}\left(Y_{1}^{\prime }\right)=Y_{1}^{\prime }*K_{4}. \end{array}$$

In our model, SCNet is used to replace the convolutional 2D convolution, which considers the context around each spatial location, avoids the information irrelevant to the lesion partly, and also improves the recognition accuracy of lung cancer lesions.

## 3. Experiments

### 3.1. Evaluation Metrics

To evaluate the performance of the proposed SC-Dynamic R-CNN on the image data that we have, we utilize a set of prevalent performance metrics for object detection, which are AP_50_, AP_75_, and mAP. AP_50_ and AP_75_ are average precision with IoU (intersection over union) thresholds of 50% and 75%. The mAP is mean average precision. The reason to choose more than one threshold is to eliminate possible evaluation biases and provide more objective evaluation results. We have partitioned our data into three groups, namely, training set, validation set, and test-dev set. The proposed Dynamic R-CNN variant is trained and validated with the training set and validation set.

The final results are reported on the test-dev set. It is worth noting that our mAP averages AP_50_ and AP_75_ for each category as a whole. Generally speaking, the better the detection effect of the model, the higher the value of mAP.

### 3.2. Implementation Details

For truthful comparisons, all experiments are implemented using PyTorch and mmdetection [37]. And the experiments are carried out in the operating environment of Ubuntu 16.04 OS with 6 ×Intel(R) Core(TM) i7-7700 CPU, using an NVIDIA GeForce RTX 2080 GPU for training. The test experiments use the same configuration. The input image size of each network is 512 × 512 pixels unless noted. We train detectors with 12 epochs with an initial learning rate of 0.01. The SGD momentum is set to be 0.9, and weight decay is with a value of 0.0001. All other hyperparameters follow the settings in mmdetection [37] if not specifically noted.

The article "SC-Dynamic R-CNN: A Self-Calibrated Dynamic R-CNN Model for Lung Cancer Lesion Detection" was published in 2022. Journal: Comput Math Methods Med.

### 3.3. Main Results

In the experimental results of this paper, we used “Adenocarcinoma,” “Squamous,” and “small cell,” to represent adenocarcinoma, squamous cell carcinoma, and small cell carcinoma, respectively.

The detection results obtained under different models are shown in the following table:

There are five contemporary methods used to compare and benchmark the results of our proposed SC-Dynamic R-CNN. The five methods are ReinaNet [21], SSD [38], Faster R-CNN [23], Libra R-CNN [27], and Cascade R-CNN [25]. These methods are among the most popular object detection neural network algorithms. The same lung cancer image data, training set, validation set, and test-dev set are used for a fair comparison. The performance of our proposed methods against the five popular methods is presented in Table 1.

The result shows that SC-Dynamic R-CNN achieves 88.1% mAP with ResNet-50, which is 8 points higher than the FPN-based Faster R-CNN baseline. As a one-stage detection network, RetinaNet and SSD achieved 81.5% and 78.9% mAP, respectively, whose accuracy is inferior to our method.

Moreover, SC-Dynamic R-CNN is much better than other networks at AP_75_. This is because SC-Dynamic R-CNN can train better results by constantly increasing the IoU threshold. Although Cascade R-CNN also achieves good results in detection, our network is higher than Cascade R-CNN no matter being at AP_50_ or AP_75_ and our mAP is 4.1 points higher than that of Cascade R-CNN.

Our proposed method demonstrates a decent level of effectiveness and robustness. The performance accuracy of our method is consistent even with different IoU thresholds. The reason why our method surpasses other methods in term of accuracy is due to the novel enhancement implemented in the previous Dynamic R-CNN algorithm. During the training phase, the proposed variant is able to automatically adjust the label assignment criteria and the shape of regression loss function so that the training set is better utilized. Another distinctive improvement is to integrate self-calibration mechanism to the RPN of the previous methods and it helps CNN generate more discriminative representations and ultimately enhances the overall performance of the variant.

The article "SC-Dynamic R-CNN: A Self-Calibrated Dynamic R-CNN Model for Lung Cancer Lesion Detection" was published in 2022. Journal: Comput Math Methods Med.

### 3.4. Ablation Experiment

To show the effectiveness of each proposed component, we report the overall ablation studies in Table 2.

These results show the effectiveness and robustness of our method.

1. DBS L1 loss: compared with Dynamic R-CNN, DBS L1 loss improves the mAP of lung cancer detection from 85.4% to 87.1%. This proves that our proposed module has better performance than the Dynamic R-CNN loss module. Results in higher IoU metrics like AP_75_ are hugely improved, which validates the effectiveness of changing the loss function to compensate for the high-quality samples during training
2. SCNet: when we replace the traditional convolution with SCNet, the mAP of lung cancer detection is improved from 87.1% to 88.1%. Compared with Dynamic R-CNN with DBL L1 loss, AP_50_ and AP_75_ increased by 0.9 points and 1.1 points, respectively, after adding SCNet. This also proves the effectiveness of SCNet for lung cancer detection

The experimental results of SC-Dynamic R-CNN are shown in the following figure:

As shown in Figure 6, this paper used the SC-Dynamic R-CNN model to detect lung cancer lesions and achieved good results. This fully demonstrates that our proposed model has greatly improved the recognition effect of lung cancer lesions.

## 4. Conclusion

To solve the problem that the biological characteristics of lung cancer were complex and difficult to detect, we proposed the SC-Dynamic R-CNN network. First, we extended the lung cancer dataset with the oversampling method and obtained the balanced dataset. Then, we added the self-calibrated convolution module to the Dynamic R-CNN network and proposed a new regression loss function, DBS L1 loss. This algorithm solves the problem of false detection and miss detection to a certain extent and greatly improves the detection accuracy of lung cancer. After experimental verification, the new algorithm achieves 88.1% mAP on the lung cancer dataset and it performed particularly well on high IoU threshold (such as AP_75_). In the next work, we will try to further improve the accuracy of the network and verify the broad applicability of the model in cancer detection.

In future, it is always worthwhile to solve this issue with some other intelligence algorithms and the bio-inspired computational methods, such as monarch butterfly optimization (MBO) [39], earthworm optimization algorithm (EWA) [40], elephant herding optimization (EHO) [41], moth search (MS) algorithm [42], slime mould algorithm (SMA) [43], hunger games search (HGS) [44], Runge Kutta optimizer (RUN) [45], colony predation algorithm (CPA) [46], Harris hawks optimization (HHO) [47], and Spiking neural P(SN-P) systems with learning [48].

The article "SC-Dynamic R-CNN: A Self-Calibrated Dynamic R-CNN Model for Lung Cancer Lesion Detection" was published in 2022. Journal: Comput Math Methods Med.

## Figures and Tables

**Figure 1:** The distribution of lung cancer CT image data of different types.

**Figure 2:** The transaxial view of the enhanced lung cancer image data.

**Figure 3:** The overall structure of the proposed SC-Dynamic R-CNN.

**Figure 4:** The curves for (a) loss and (b) gradient of our regression loss with different *α*. *α* is set to default as 1.0.

**Figure 5:** The overall structure of SCNet.

**Figure 6:** SC-Dynamic R-CNN detection effect diagram. Adenocarcinoma test results (left), small cell carcinoma test results (center), and squamous carcinoma test results (right).

**Table 1:** Comparisons with different models on our lung cancer dataset.

Method	Backbone	Adenocarcinoma		Squamous		Small cell		mAP
		AP_50_	AP_75_	AP_50_	AP_75_	AP_50_	AP_75_	
RetiNanet [21]	ResNet-50	87.7%	67.8%	89.7%	79.9%	88.1%	77.8%	81.8%
SSD [38]	ResNet-50	80.7%	61.4%	89.2%	78.4%	86.2%	77.3%	78.9%
Faster R-CNN [23]	ResNet-50	81.6%	62.5%	90.5%	80.3%	89.7%	79.4%	80.1%
Libra R-CNN [27]	ResNet-50	81.9%	71.4%	89.9%	81.5%	89.3%	83.2%	82.9%
Cascade R-CNN [25]	ResNet-50	82.7%	73.5%	90.1%	82.9%	90.1%	84.9%	84.0%
SC-Dynamic R-CNN	ResNet-50	**91.6%**	**77.3%**	**91.5%**	**88.2%**	**91.4%**	**88.6%**	**88.1%**

**Table 2:** Results of each component in SC-Dynamic R-CNN on val set.

Backbone	FPN	DBS L1 loss	SCNet	AP50	AP75	mAP
ResNet-50	√			90.1%	80.7%	85.4%
ResNet-50	√	√		90.6%	83.6%	87.1%
ResNet-50	√	√	√	91.5%	84.7%	88.1%

## Data Availability

The data can be provided upon request.
